# Effect of Core Stability Training on Unstable Support Surfaces in Postoperative Rehabilitation of Thoracolumbar Vertebral Compression Fractures in the Elderly

**DOI:** 10.1155/2022/4480349

**Published:** 2022-10-17

**Authors:** Yanfei Yin, Shixia Cao, Chenjie Wang, Yanju Liu, Huakai Zhang

**Affiliations:** ^1^Department of Rehabilitation Teaching and Research, Medical College of Zhengzhou University of Industrial Technology, Xinzheng, Henan 451100, China; ^2^Department of Rehabilitation Medicine, South Branch of the First Affiliated Hospital of Zhengzhou University, Zhengzhou, Henan 450000, China

## Abstract

**Objective:**

Thoracolumbar vertebral compression fractures (TVCF) are caused by anterior flexion or vertical downward violence to the spine (Sezer et al. 2021). This study is aimed at investigating the effect of core stability training (CST) on unstable support surfaces in the postoperative rehabilitation of TVCF in the elderly*. Methods*. Ninety-eight patients with TVCF who underwent surgical treatment in our hospital from July 2021 to April 2022 were selected as study subjects. Then, they were divided into a research group receiving unstable support surface CST and a control group with conventional rehabilitation training according to the random number table method. Before and after the training, the X-ray machine was positioned and the anterior margin and middle height ratio and the posterior convex Cobb angle of the injured vertebrae were observed, and the balance detector was used to detect patients' eye opening and closing trajectory length, Romberg rate, and to perform gait test. Patients' pain, lumbar spine function, and quality of life were subsequently assessed using the Visual Analogue Scale (VAS), Oswestry Dysfunction Index (ODI), Generic Quality of Life Inventory-74 (GQOL-74), and patient satisfaction with rehabilitation was investigated*. Results*. After rehabilitation training, there was no statistically marked difference in eye-opening trajectory length between both groups (*P* > 0.05). The research group had higher scores than the control group in all dimensions of the anterior border of the injured vertebra, middle height ratio, and GQOL-74, while the posterior convex Cobb angle, closed-eye trajectory length, Romberg rate, VAS, and ODI were lower than the control group (*P* < 0.05). The research group also revealed better gait improvement and higher rehabilitation satisfaction than the control group after training (*P* < 0.05).

**Conclusion:**

Unstable support surface CST can effectively improve postoperative vertebral body rehabilitation, balance function, gait, pain conditions, and lumbar spine function in elderly TVCF patients, and enhance their quality of life and rehabilitation satisfaction. This trial is registered with ChiCTR2000014547.

## 1. Introduction

Thoracolumbar vertebral compression fractures (TVCF) are caused by anterior flexion or vertical downward violence to the spine [1]. It is also prone to occur in middle-aged and elderly people, where osteoporosis leads to reduced bone mass, decreased strength, and increased fragility of the cone, and is also a high-risk factor for TVCF [2]. Statistics show that on average, more than 600,000 new cases of TVCF are diagnosed each year worldwide, and they are predominantly female [3]. TVCF are mainly occurring in the lower thoracic and upper lumbar segments. The clinical manifestations were back pain and cannot move, which could hinder standing and walking. If compression is severe, the spinous process or ligaments of the posterior column may be damaged, resulting in local kyphosis, swollen ecchymosis, or neurological symptoms such as lower limb numbness and urinary and fecal incontinence, which seriously affect the normal life of patients [4]. Currently, conservative treatment of clinically targeted TVCF is time-consuming and prolonged bed rest increases the incidence of complications such as pressure sores and lower extremity venous thrombosis [5]. Therefore, most patients choose surgical treatment to solve their pain as soon as possible. But due to the reduced muscle function and poor physical tolerance of elderly patients, the recovery after surgery has been unsatisfactory, and in more serious cases, surgery may cause more serious spinal complications [6, 7]. Therefore, a method that can effectively enhance the postoperative recovery of TVCF patients has also been searched for in the clinical practice.

Recently, the application of postoperative rehabilitation exercises after surgical treatment of various diseases has attracted clinical attention. Researchers have found that rehabilitation exercises can not only effectively improve the pathological recovery process of patients but also enhance their organism function and improve their prognostic quality of life [8]. Currently, postoperative rehabilitation exercises have achieved excellent application results in the treatment of stroke and heart failure [9, 10]. Among them, core stability training (CST) is one of the effective physical training methods promoted in recent years and has been gradually introduced into the field of rehabilitation medicine, which can effectively improve the body's coordinated control of various parts of the muscles [11]. As reported previously, CST can improve chronic spinal cord injury patients' ambulation and static balance function [12]. Besides, CST can be used as an efficient clinical intervention to improve dynamic and static balance and core muscle function in women with multiple sclerosis [13]. The unstable support surface CST, on the other hand, accelerates the promotion of balance and stability of patients' organism through unstable support, enhances the control of muscle movement, and helps the recovery of limb function [14]. At the moment, unstable support surface CST has been shown to be effective in improving limb movement function in stroke patients [15], but the effectiveness of its application in TVCF is not yet known.

We believe that unstable support surface CST may also have a remarkable enhancement effect on postoperative rehabilitation of elderly TVCF. Thus, to confirm the conjecture and expect to provide effective reference for the future clinical treatment of TVCF, the effect of unstable support surface CST in postoperative rehabilitation of TVCF in the elderly will be investigated.

## 2. Materials and Methods

### 2.1. Patient Data

Ninety-eight patients with TVCF in our hospital from July 2021 to April 2022 were selected as the study population. Among these, 49 patients with 30 males and 19 females, and mean age was 65.10 were divided into the control group. 49 patients with 28 males and 21 females, and mean age was 64.47 were divided into the research group. Inclusion criteria are as follows: (1) complete clinical data; (2) clinical diagnosis of TVCF [16] and completion of surgical treatment in our hospital. (3) age>60 years old; (4) no spinal cord compression; (5) no nerve root injuries; and (6) patients agree and are willing to participate in rehabilitation therapy. Exclusion criteria are as follows: (1) combined with other osteoarticular diseases; (2) presence of cognitive impairments; (3) low compliance with treatment; and (4) patients who stopped the trial early for other reasons. The patients were divided into research and control groups according to the random number table method. Patients in the research group were given unstable support surface CST, and the control group was given conventional rehabilitation training. The study was conducted in strict compliance with the Declaration of Helsinki and was approved by the Ethics Committee of our hospital. All study subjects signed an informed consent form by themselves.

### 2.2. Training Methods

Control group is as follows: (1) turning training: the responsible nurse began to instruct and assist the patients to turn over 12 h after surgery, helping them to straighten the waist and back, turning over once every 2 h, and trying to let them finish turning over independently after 48 h. (2) Postural training: 7 d after training, abdominal jerk training was started, 15 min/time, 6 times/d. (3) Lower limb training: 24 h after training, the responsible nurse instructed the patients to carry out leg raising exercises and ankle rotation exercises, alternately raising both lower limbs and holding them up for 5 s, and slowly lowering them, 15 min/time, 5 times/d. (4) For functional training of the lumbar back muscles, after 14 d of training, patients performed five-point support training of both feet, both axes and head, which was replaced with three-point support training of both feet and head after 21 d, 5 s/time, 10 times/d. (5) Dietary guidance: low-salt, high-calcium foods such as fish, bone broth, and eggs were the mainstay, and vitamin D and calcium supplements were reinforced. (6) Antiosteoporosis treatment: oral treatment with calcium carbonate D3 tablets (2 times/d) and intravenous zoledronic acid injection (5 mg/d, 1 time/d) for a period of 3 months. Research group: unstable support surface CST [12] was carried out with reference to the study of Liu et al. (1) Bridge exercise: patients were in the supine position, putting the proximal ends of both lower legs into the suspension rope, raising the buttocks, extending the hips, maintaining the trunk, knee, shoulder, and hip joints in the same line, each time for 10 s. (2) Plank support: patients lied prone, bended both elbows to support the bed, set the proximal ends of both calves into the suspension rope, left the body off the bed, ensuring that the ankle, hip, shoulder, and head to remain in a straight line, tightening the abdominal muscles and pelvic floor muscles, and lengthening the spine for 10 s. (3) Lateral plate support: patients lied on his side, supported by the foot and unilateral elbow joint on the bed, with the proximal ends of both lower legs set into the suspension rope, keeping the lower limbs, trunk and head off the bed in a straight line for 10 s. (4) Sitting training: patients sat on a therapy ball with the pelvis tilted forward and backward to keep the upper trunk stable. They lifted one side of the pelvis and sat to keep the upper trunk stable. Rotating both knees back and forth and keeping the upper trunk stable in the seated position. Lateral bending at the waist, unilateral elbow down, keeping the upper trunk stable. Each movement lasted 5 s in the seated position. The above training movements were performed with the assistance of a therapist, using an elastic suspension device for weight loss assistance, if necessary, for 30 min each time, 1 time/d, 5 times/week, for 8 weeks. (5) Dietary guidelines: same to the control group. (6) Antiosteoporosis treatment: same to the control group.

### 2.3. Outcome Measures

The outcome measures are as follows. (1) Vertebral rehabilitation: the patients were placed in a prone position with padding of the chest, both shoulders, and the anterior superior iliac spine, keeping the spine in a hyperextended position, using a C-arm X-ray machine to locate and observe the anterior margin, middle height ratio, and posterior convex Cobb angle of the injured vertebra. The greater the height ratio of the injured spine, the smaller the value of the posterior convexity Cobb angle indicating better recovery of the injured spine. (2) Balance function: it was assessed using a balance tester (Active Balance EAB-100, Sakai, Japan). The patient naturally separated his feet after taking off his shoes and stood parallel with his hands hanging down naturally to maintain stability. Open-eye and closed-eye tests were conducted separately for 1 min each with an interval of 30 s. The track length and Romberg rate were recorded, and the smaller the value, the better the stability. (3) Gait: use the meter ruler to measure and record the stride length, the number of strides in 1 min, and the distance of each step in a comfortable state, the higher the value, the better the gait. (4) Routine scoring: patients were assessed for pain using a visual analogue scale (VAS) [17] with a 10 cm long vernier scale with 10 scales on one side and “0” and “10” scales at each end, with 0 indicating no pain and 10 indicating the most severe pain that is unbearable. Lumbar spine function was assessed using the Oswestry Dysfunction Index (ODI) [18], which consists of 10 questions with 6 options for each question and a maximum score of 5, with higher scores indicating poorer lumbar spine function. Patients' quality of life was assessed using the Generic Quality of Life Inventory-74 (GQOL-74) [19], which includes 4 dimensions of psychological function, physical function, material life, and social function, the score of each dimension was 0-100, with higher scores indicating better quality of life. (5) Rehabilitation satisfaction: after patients' rehabilitation training was completed, a survey on rehabilitation satisfaction was conducted using our homemade scale statistics, and the results were classified as very satisfied, basically satisfied, and dissatisfied. Total satisfaction = (very satisfied + basically satisfied)/total number of people × 100%.

### 2.4. Statistical Methods

Statistical analysis was performed using SPSS 23.0 software, with the counting data expressed as (*n* (%)) and the chi-square test used for comparison between groups. The measurement data were represented as ($\bar{x}\pm s$), and independent sample *t*-test was used for comparison between groups, and paired *t*-test was used for intragroup comparison before and after treatment. *P* < 0.05 indicates that the difference is statistically remarkable.

## 3. Results

### 3.1. Comparison of Clinical Baseline Data

To ensure the credibility of the experimental results, we first compared the baseline data such as age, BMI, course of osteoporosis, gender, type of injury, smoking, and drinking between both groups. It was seen that none of the differences were statistically remarkable (*P* > 0.05), confirming that both groups were comparable (Table 1).

### 3.2. Comparison of Vertebral Body Rehabilitation

Before training, there was no statistically remarkable difference between both groups in the anterior and middle height ratios of the injured spine and the posterior convex Cobb angle (*P* > 0.05). While after training, the anterior and middle height ratios of the injured spine increased in both groups and were higher in the research group than in the control group (*P* < 0.05), while the posterior convex Cobb angle was decreased in both groups and was lower in the research group compared to the control group (*P* < 0.05) (Figure 1).

### 3.3. Comparison of Balance Function

Before training, the eye-opening and closed-eye trajectory length and Romberg rate of both groups were also not dramatically different (*P* > 0.05), while after training, the eye-opening and closed-eye trajectory length and Romberg rate of both groups were lower than those before treatment (*P* < 0.05). Among them, no difference was found between the research group and the control group in the open-eye trajectory length (*P* > 0.05), but the closed-eye trajectory length and Romberg rate in the research group were both lower than those of the control group (*P* < 0.05) (Figure 2).

### 3.4. Comparison of Gait

There were no statistically remarkable differences between the research group and control group in terms of stride length, number of strides within 1 min, and distance per step in a comfortable state before training (*P* > 0.05). However, the stride length, the number of strides in 1 min, and the distance per step in a comfortable state were dramatically improved in both groups after training compared with those before training (P <0.05), while the gait indexes of the research group were all higher than those of the control group after training (P <0.05). (Figure 3).

### 3.5. Comparison of Pain Conditions and Lumbar Spine Function

Similarly, it was seen that there was no marked difference in VAS scores and DOI between the research and control groups before training (*P* > 0.05) and VAS scores and DOI were dramatically lower in both groups after training (*P* < 0.05). However, the VAS scores and DOI after training were lower in the research group than in the control group (*P* < 0.05) (Figure 4).

### 3.6. Comparison of Quality of Life

It was seen that the scores of psychological functions, physical function, material life, and social function were higher in the research group than in the control group (*P* < 0.05) (Figure 5).

### 3.7. Comparison of Rehabilitation Satisfaction

The results of the satisfaction survey denoted that only 3 patients in the research group was dissatisfied with the rehabilitation, and the total satisfaction reached 93.88%, while the total satisfaction of the control group was only 77.55%. The total satisfaction of the research group was higher than that of the control group (*P* = 0.021) (Table 2).

## 4. Discussion

It is well known that the lumbar and thoracic spine are the core parts of the body that maintain upright walking and are also the parts that remain stable during exercise [20, 21]. Core stability refers to the ability of the trunk and pelvis to play a stable posture in human movement, which can effectively control the center of gravity, coordinate upper and lower limbs to generate, and control and transmit power [22]. Thus, CST can help build a strong core muscle group, which in turn can influence the dynamic chain function of the organism [23]. Besides, it has also been found that some specific core muscles are activated throughout the gait cycle by surface EMG probing, which also suggests that CST practice is important for walking rehabilitation [24]. With the serious problem of aging population, TVCF has also become higher. Although symptoms can be relieved to a certain extent in clinical practice after surgical treatment such as percutaneous vertebroplasty is given, postoperative rehabilitation exercises are still needed to restore limb function as soon as possible [25, 26]. Hence, this study is important for the future treatment of TVCF regarding the effect of unstable support surface CST on the rehabilitation outcome of patients.

It showed that patients in the research group had more obvious improvement in vertebral rehabilitation, balance function, gait, and lumbar spine function after CST with an unstable support surface than the control group, suggesting that our CST with an unstable support surface can be more effective in improving postoperative rehabilitation of TVCF patients. In previous studies, unstable support surface CST has also been found to facilitate the rehabilitation process of hip arthroplasty patients, improving gait, balance, and coordination [27]. This can also corroborate the results of the current experiment. We believe that patients have facilitated the functional recovery of the muscle groups through the unstable support surface CST, and they are able to obtain protection during exercise similar to the corset effect and are able to perform better motor transmission with this effective muscle strength [28]. In the meantime, patients were trained in non-steady-state conditions, constantly changing various postures, and looking for a state to control their own center of gravity and ensure body balance. It helps the body's nerve tissue to effectively control balance, also improves muscle strength, and promotes the body's balance and stability [29]. However, there was no difference in the length of the open-eye trajectory between both groups after CST with an unstable support surface in the balance examination. We speculate that this may be because in the open-eye state, both patients could better maintain their balance. In the closed-eye state, the control group patients lost visual aids and therefore had less control over the organism, while the research group, which had better control over the organism, revealed more excellent balance ability. In addition, we found that VAS scores and DOI after training were lower in the research group than in the control group, suggesting that patients with unstable support surface CST had less pain than those with conventional rehabilitation training. Consistently, previous literature has indicated that CST can alleviate pain in patients with chronic nonspecific low back pain [30]. Combined with relevant studies in rehabilitation medicine [31–34], we concluded that the improvement of limb coordination and control by CST on unstable support surfaces was specifically achieved through the following points: (1) bridge exercises can help control lower extremity extensor spasm conditions, improve pelvic coordination, and control of the lower extremities, and help patients stand and walk. (2) Plank support is a muscle training similar to push-ups, without the up and down support movement, the patient takes a prone position, keeping the main body parts in a straight line, which can effectively exercise the transverse abdominal muscles, enhance trunk muscle control, and provide support for upper and lower limb movement. (3) The right lateral plank support can help improve pelvic control, which in turn provides adequate support for lower body movements. (4) The training of the pelvis, knees, waist, shoulders, and hands is carried out with the help of therapy balls in the sitting training, which can effectively balance the movement of all parts of the body and promote the coordination of the body. (5) The length of the musculotendinous complex determines the speed and size of the gait. Further investigation revealed that the unstable support surface increased muscle tone contractility through the trained tonic vibration reflex, which in turn enhanced trunk control through proprioception, and thus patients' walking speed and stride length were dramatically higher. Combining these positive effects, the unstable support surface CST was more effective in enhancing the postoperative recovery of TVCF patients, which we believe is the main reason for the better quality of life after training in the research group. In previous studies, we have also found that unstable support surface CST improves the prognostic quality of life in patients with chronic low back pain [35], again corroborating our view that the scores of psychological functions, physical function, material life, social function in patients with unstable support surface CST were higher than those with conventional rehabilitation training. Furthermore, patient satisfaction naturally increases as the recovery is optimized, which together again emphasizes the future value of the unstable support surface CST for excellent clinical applications.

Nevertheless, there is still a lack of uniform clinical guidelines for unstable support surface CST in clinical practice. Thus, there may be room for improvement and optimization of the rehabilitation training content implemented in this study. Also, due to the short follow-up period, it is vague what the long-term prognostic impact of unstable support surface CST is on patients. What's more, the effect monitoring indexes selected in this study are relatively limited, and further observations and comparisons can be made by ultrasound and biofeedback analysis system on the trunk muscle thickness and central sway area of patients to obtain more comprehensive results for clinical reference.

## 5. Conclusion

Unstable support surface CST can effectively improve postoperative vertebral body rehabilitation, balance function, gait, pain conditions, and lumbar spine function in elderly TVCF patients, and enhance their quality of life and rehabilitation satisfaction. Hence, it is of great value in clinical applications.

## Figures and Tables

**Figure 1:** Comparison of vertebral body rehabilitation. (a) Height ratio of the anterior margin of the injured spine before and after training in both groups. (b) Height ratio of the middle of the injured spine before and after training in both groups. (c) Two sets of training before and after the posterior convex Cobb angle. # indicates that the difference is statistically significant compared with before training (*P* < 0.05). & indicates that the difference is statistically significant compared with the control group (*P* < 0.05).

**Figure 2:** Comparison of balance function. (a) The eye-opening trajectory was long before and after the two sets of training. (b) The closed-eye trajectory was long before and after two sets of training. (c) Romberg rate before and after training in both groups. # indicates that the difference is statistically significant compared with before training (*P* < 0.05). & indicates that the difference is statistically significant compared with the control group (*P* < 0.05).

**Figure 3:** Comparison of gait. (a) Two sets of training front and back stride length. (b) Number of strides in 1 min before and after the two sets of training. (c) Distance per step in the comfortable state before and after the two sets of training. # indicates that the difference is statistically significant compared with before training (*P* < 0.05). & indicates that the difference is statistically significant compared with the control group (*P* < 0.05).

**Figure 4:** Comparison of pain conditions and lumbar spine function. (a) Comparison of VAS scores. (b) Comparison of DOI. # indicates that the difference is statistically significant compared with before training (*P* < 0.05). & indicates that the difference is statistically significant compared with the control group (*P* < 0.05).

**Figure 5:** Comparison of quality of life. (a) Comparison of psychological functions scores. (b) Comparison of physical function scores. (c) Comparison of material life scores. (d) Comparison of social function scores. # indicates that the difference between the two groups is statistically significant (*P* < 0.05).

**Table 1:** Clinical baseline data.

	Age	BMI (kg/m^2^)	Course of osteoporosis (years)	Gender male/female	Type of injury 6-12 thoracic/1-5 lumbar	Smoking yes/no	Drinking yes/no
Control group (*n* = 49)	65.10 ± 5.41	23.52 ± 4.23	4.39 ± 1.86	30/19	22/27	26/23	18/31
Research group (*n* = 49)	64.47 ± 5.26	24.14 ± 5.50	4.20 ± 1.66	28/21	25/24	25/24	21/28
*t* or *χ*^2^	0.584	0.626	0.534	0.169	0.368	0.041	0.383
*P*	0.560	0.533	0.595	0.681	0.544	0.840	0.536

**Table 2:** Rehabilitation satisfaction.

	Very satisfied	Basically satisfied	Dissatisfied	Total satisfaction (%)
Control group (*n* = 49)	22 (44.90)	16 (32.65)	11 (22.45)	77.55
Research group (*n* = 49)	31 (63.27)	15 (30.61)	3 (6.12)	93.88
*χ* ^2^				5.333
*P*				0.021

## Data Availability

The datasets used and/or analyzed during the current study are available from the corresponding author on reasonable request.
